RETRACTED

# The Clinical Effect of High-Flow Oxygen Therapy through the Nose on Patients with Acute Left Heart Failure and Hypoxemia

**DOI:** 10.1155/2022/7117508

**Published:** 2022-03-14

**Authors:** Xinlei Hao, Shuoran Zhao, Jiajia Cheng, Lihua Yang, Haiming Jiang, Fuzheng Qu

**Affiliations:** ^1^Department of Critical Care Medicine, Yantai Affiliated Hospital of Binzhou Medical University, Yantai 264100, Shandong, China; ^2^Department of Cardiovascular Medicine, Yantai Affiliated Hospital of Binzhou Medical University, Yantai 264100, Shandong, China

## Abstract

**Objective:**

To evaluate the clinical efficacy of nasal high-flow oxygen therapy in patients with acute left heart failure and hypoxemia.

**Methods:**

From July 2016 to November 2018, patients with acute left heart failure complicated with hypoxemia treated in the Department of Critical Medicine of Yantai Affiliated Hospital of Binzhou Medical University were retrospectively observed (a total of 140 cases met the inclusion criteria). They were randomly divided into two groups, with 70 cases in each group. Patients were given continuous ECG monitoring, improved blood gas analysis test, and recorded HR, RR, map, SaO_2_, pH, PaO_2_, PaCO_2_, and Lac, perfect examination and color Doppler echocardiography, and record NT-proBNP and EF before and 24 hours after treatment. The effective rates of the two groups before and after oxygen therapy were detected.

**Results:**

There were 67 patients with high-flow oxygen therapy group improvement, 95.7% improvement rate, and 55 patients with general oxygen therapy group improvement rate. The treatment improvement rate was 78.6%. A total of 67 patients were treated with high-flow oxygen therapy. After high-flow oxygen therapy, HR (*t* = 18.8, *P* ≤ 0.05), RR (*t* = 19.7, *P* ≤ 0.05), MAP (*t* = 12.1, *P* ≤ 0.05), PaCO_2_ (*t* = 9.53, *P* ≤ 0.05), Lac (*t* = 8.69, *P* ≤ 0.05), and NT-proBNP (*t* = 7.03, *P* ≤ 0.05) were significantly lower than before. SaO_2_ (*t* = −12.4, *P* ≤ 0.05), pH (*t* = −12.2, *P* ≤ 0.05), PaO_2_ (*t* = −17.7, *P* ≤ 0.05), and EF (*t* = −13.4, *P* ≤ 0.05) were significantly higher than before. A total of 55 patients were in the general oxygen therapy group. After administration of ordinary oxygen therapy, HR (*t* = 18.2, *P* ≤ 0.05), RR (*t* = 10.8, *P* ≤ 0.05), MAP (*t* = 13.1, *P* ≤ 0.05), PaCO_2_ (*t* = 15.8, *P* ≤ 0.05), Lac (*t* = 7.1, *P* ≤ 0.05), and NT-proBNP (*t* = 10, *P* ≤ 0.05) were significantly lower than before. SaO_2_ (*t* = −15.5, *P* ≤ 0.05), pH (*t* = −4.5, *P* ≤ 0.05), PaO_2_ (*t* = −20, *P* ≤ 0.05), and EF value (*t* = −7.7, *P* ≤ 0.05) were significantly higher than before.

**Conclusion:**

High-flow oxygen therapy and general oxygen therapy have an obvious curative effect on patients with acute left heart failure and hypoxemia. Compared with the two, high-flow oxygen therapy is more effective. After high-flow oxygen therapy and general oxygen therapy in patients with acute left heart failure and hypoxia, HR, RR, MAP, SaO_2_, pH, PaO_2_, PaCO_2_, Lac, EF, and NT-proBNP value all improved, and the improvement of high-flow oxygen therapy was greater.

RETRACTED

## 1. Introduction

Cardiovascular disease has become the primary problem threatening human health. Heart failure is an important part of cardiovascular disease that cannot be ignored. If acute heart failure occurs or the basic state is poor, the prognosis is often poor. In recent years, with the vigorous development of medical research, the diagnosis of heart failure has become more precise, the treatment methods have become more abundant, and the treatment effect has become more significant. As a commonly used treatment method, oxygen therapy has always played an important role in the adjuvant treatment of critically ill patients. Patients with acute left heart failure often have restrictive hypoventilation and diffuse dysfunction. Actively correcting hypoxemia and improving respiratory status as soon as possible can improve the therapeutic effect of heart failure. On the basis of conventional medical treatment, the application of assisted respiratory support is for the treatment of heart failure, the main goal of which is to maintain the oxygen supply of the tissues, relieve symptoms as soon as possible, and improve the prognosis. At present, the conventional oxygen therapy methods include nasal catheter oxygen inhalation and mask oxygen inhalation, but the effect is general. The application of high-flow oxygen therapy has previously focused on neonatal and respiratory diseases, but not much involved in circulatory diseases. The aim of this study was to evaluate the clinical efficacy of nasal high-flow oxygen therapy in patients with acute left heart failure and hypoxemia. The clinical efficacy will provide a certain theoretical basis for the future treatment of this disease with high-flow oxygen therapy.

## 2. Object and Methods

### 2.1. Research Object

1. A randomized controlled trial was conducted to collect 140 patients with acute left heart failure complicated with hypoxemia treated in Yantai Affiliated Hospital of Binzhou Medical University from July 2016 to November 2018, including 89 male patients (63.6%) and 51 female patients (36.4%); all patients were aged 43–96 years, with an average of 70.75 years. Inclusion criteria: meet the diagnostic criteria for acute left heart failure in the eighth edition of internal medicine (dyspnea, orthopedic breathing, cyanosis of the lips, profuse sweating, and coughing up a lot of pink foamy sputum; both lungs are symmetrically filled with wet rales; BNP or NT-ProBNP increased) and meet the diagnostic criteria for hypoxemia (Arterial partial pressure of oxygen (PaO_2_) is lower than the lower limit of normal for people of the same age, and the calculation formula for different ages: oxygen partial pressure = 100–0.3 *∗* age ± 5 mmHg) [1]. Exclusion criteria: patients who cannot accept and cooperate with high-flow oxygen therapy, patients with severe renal insufficiency (creatinine >133 umol/L) [2], and patients with unstable hemodynamics. Using a random number table, the patients were numbered according to the time of visit and admission, and the patients were divided into two groups, a control group and an experimental group, with 70 cases in each group. Their age, gender, comorbidities, and ejection fraction were statistically analyzed. The above difference is not significant (Table 1). This study was approved by the Yantai Affiliated Hospital of Binzhou Medical University Ethics Committee, and all patients signed the informed consent.

RETRACTED

### 2.2. Oxygen Therapy Methods

Under the same conditions as other general drugs (cardiotonic, diuretic, and vasodilator), the control group was given ordinary oxygen therapy (mask (flow rate 6–10 L/min) or nasal catheter oxygen inhalation (flow rate 3–5 L/min)). The experimental group was given transnasal high-flow oxygen therapy (flow rate 10–60 L/min).

### 2.3. Observation Indicators

1. Judgment of the curative effect: effective: symptoms improved, vital signs such as heart rate, respiration, and blood pressure gradually stabilized, and arterial blood gas indicators improved. Invalid: not up to the above standards.
2. Monitor and record the changes of HR, RR, MAP, SaO_2_, pH value, PaO_2_, PaCO_2_, Lac, NT-proBNP, EF value, and other indicators before and after the use of different oxygen therapy methods.

### 2.4. Statistical Methods

The SPSS 23.0 statistical software package was used for statistical processing. The normality test of measurement data adopts the K-S method. Normally distributed data are expressed as mean ± standard deviation ($\bar{x}\pm s$), using the *t* test. *P* < 0.05 was considered to be a significant difference.

## 3. Results

### 3.1. Comparison of the Effective Rates of the Two Treatments

A total of 140 patients with acute left heart failure and hypoxemia were included in the trial. The experimental group (high-flow oxygen therapy group) consists of 70 cases, of which 67 cases were effective in treatment, and the effective rate was about 95.7%; the control group (normal oxygen therapy group) consists of 70 cases, of which 55 cases were effective, and the effective rate was about 78.6%, as given in Table 2)

RETRACTED

### 3.2. Changes of Indicators in the High-Flow Oxygen Therapy Group before and after Treatment

There were 67 effective patients in the high-flow oxygen therapy group. The HR, RR, MAP, SaO_2_, pH value, PaO_2_, PaCO_2_, and Lac were recorded before and 2 hours after the high-flow oxygen therapy, EF value, and NT-proBNP value. The results of statistical analysis showed the following: HR (*t* = 18.8, *P* ≤ 0.05), RR (*t* = 19.7, *P* ≤ 0.05), MAP (*t* = 12.1, *P* ≤ 0.05), and PaCO_2_ (*t* = 9.53, *P* ≤ 0.05) of patients after high-flow oxygen therapy; Lac (*t* = 8.69, *P* ≤ 0.05) and NT-proBNP (*t* = 7.03, *P* ≤ 0.05) were significantly lower than before. SaO_2_ (*t* = −12.4, *P* ≤ 0.05), pH value (*t* = −12.2, *P* ≤ 0.05), PaO_2_ (*t* = −17.7, *P* ≤ 0.05), and EF value (*t* = −13.4, *P* ≤ 0.05) are all significantly higher than before (Table 3).

### 3.3. Changes of Indicators in the Ordinary Oxygen Therapy Group before and after Treatment

A total of 55 patients in the ordinary oxygen therapy group were treated effectively. The HR, RR, MAP, SaO_2_, pH, PaO_2_, PaCO_2_, and Lac before and 2 hours after the treatment were recorded; the EF values before and 24 hours after the treatment are the NT-proBNP value. The results of statistical analysis showed the following: HR (*t* = 18.2, *P* ≤ 0.05), RR (*t* = 10.8, *P* ≤ 0.05), MAP (*t* = 13.1, *P* ≤ 0.05), and PaCO_2_ (*t* = 15.8, *P* ≤ 0.05) of patients after ordinary oxygen therapy; Lac (*t* = 7.1, *P* ≤ 0.05) and NT-proBNP (*t* = 10, *P* ≤ 0.05) were significantly lower than before, and the difference was statistically significant. SaO_2_ (*t* = −15.5, *P* ≤ 0.05), pH value (*t* = −4.5, *P* ≤ 0.05), PaO_2_ (*t* = −20, *P* ≤ 0.05), and EF value (*t* = −7.7, *P* ≤ 0.05) are all significantly higher than before high, and the difference is statistically significant (Table 4).

### 3.4. Comparison of the Improvement of Various Indicators before and after High-Flow Oxygen Therapy and Ordinary Oxygen Therapy

By calculating the difference between the changes of various indicators before and after treatment in the high-flow oxygen therapy group and the ordinary oxygen therapy group, statistical analysis can be seen. HR, RR, MAP, SaO_2_, pH value, PaO_2_, PaCO_2,_ Lac, EF value, and NT-proBNP value were significantly greater than that of the ordinary oxygen therapy group (Table 5).

## 4. Discussion

Hypoxemia caused by acute heart failure is a clinically critical illness, which is extremely life-threatening to patients, and immediate targeted therapeutic intervention is required to effectively control the condition [3, 4]. Under normal circumstances, the patient will have difficulty breathing, sweating, cyanosis, and coughing pink foamy sputum, and there are wet rales and wheezing in both lungs after physical examination and auscultation [5]. Clinically, some patients' condition has not been significantly improved in time after conventional (drug) treatment, and the correction of heart failure is not obvious. The subsequent circulatory disorders and the mortality rate have been significantly increased [6]. On the basis of the application of conventional drug therapy, giving a ventilator or oxygen therapy device, through the method of mechanical ventilation, quickly corrects hypoxemia, alleviates the patient's acidosis, and can more quickly correct heart failure [7].

RETRACTED

We explore the effect of high-flow oxygen therapy in patients with acute left heart failure and hypoxemia. HFNC can correct hypoxemia better and faster and improve respiratory function. Hypoxemia can be corrected by increasing oxygen flow, giving appropriate PEEP, and reducing the work of breathing of the patient, thereby improving the body's oxygen supply, reducing the damage of hypoxia to myocardial cells, alleviating symptoms, and improving heart failure [8–10]. The premise is based on the basic drug treatment that has been given to patients with heart failure, and the treatment effect is not ideal if oxygen therapy is given without drug intervention.

The study compared the therapeutic effects of high-flow oxygen therapy and ordinary oxygen therapy, but there are still many problems that need to be resolved or perfected, such as there is no clear guideline for weaning indications when weaning is still based on the experience of clinician's host. In addition, how to adjust the weaning time also has the problem of ambiguous concept [11, 12]. Although clinical studies have found that patients using high-flow oxygen therapy can effectively reduce the length of hospital stay and improve survival rate and the treatment efficiency of high-flow oxygen therapy is significantly better than ordinary oxygen therapy, there are still patients with heart failure and hypoxemia. In the case that high-flow oxygen therapy is ineffective, some studies have pointed out that when high-flow oxygen therapy fails, the intubation time of patients is significantly longer than that of the overall hospitalized patients, and the mortality rate is also significantly increased. This is also a problem worthy of our attention.

## Figures and Tables

**Table 1:** Comparison of clinical data between the two groups of patients.

Patient characteristics	Control group (*n* = 70)	Experimental group (*n* = 70)	*P* value
Age (years, *x* ± *s*)	101.19 ± 15.59	87.7 ± 15.5	*P* > 0.05
Male (composition ratio, %)	24.58 ± 3.80	18.88 ± 2.77	*P* > 0.05
Complications (composition ratio, %)	103.48 ± 16.95	88.90 ± 13.95	*P* > 0.05
Ejection fraction (%)	85.8 ± 7.35	95.72 ± 2.2	*P* > 0.05

RETRACTED

**Table 2:** Summary of the comparison of the effective rates of the two treatment methods.

Project	High-flow oxygen therapy group	Ordinary oxygen therapy group
Effective number of cases	67	55
Efficient	95.7%	78.6%

**Table 3:** Summary of changes in indicators in the high-flow oxygen therapy group before and after treatment.

Project	High-flow oxygen therapy group		*t* value	*P* value
	Before therapy	After treatment		
HR	101.19 ± 15.59	87.7 ± 15.5	18.8	*P* ≤ 0.05
RR	24.58 ± 3.80	18.88 ± 2.77	19.7	*P* ≤ 0.05
MAP	103.48 ± 16.95	88.90 ± 13.95	12.1	*P* ≤ 0.05
SaO_2_	85.8 ± 7.35	95.72 ± 2.2	−12.4	*P* ≤ 0.05
pH value	7.31 ± 0.63	7.38 ± 0.51	−12.2	*P* ≤ 0.05
PaO_2_	58.78 ± 8.48	83.24 ± 13.31	−17.7	*P* ≤ 0.05
PaCO_2_	50.51 ± 10.88	41.52 ± 7.66	9.53	*P* ≤ 0.05
Lac	3.39 ± 2.83	2.09 ± 2.09	8.69	*P* ≤ 0.05
EF value	46.21 ± 9.07	56.36 ± 5.92	−13.4	*P* ≤ 0.05
NT-proBNP	12057.61 ± 9547.99	8136.80 ± 7607.01	7.03	*P* ≤ 0.05

**Table 4:** Summary of changes in various indicators before and after treatment in the ordinary oxygen therapy group.

Project	Normal oxygen therapy group		*t* value	*P* value
	Before therapy	After treatment		
HR	91.05 ± 14.37	80.5 ± 14.02	18.2	*P* ≤ 0.05
RR	22.36 ± 4.04	19.07 ± 3.37	10.8	*P* ≤ 0.05
MAP	99.05 ± 12.97	88.33 ± 11.66	13.1	*P* ≤ 0.05
SaO_2_	86.4 ± 4.81	93.44 ± 2.98	−15.5	*P* ≤ 0.05
pH value	7.33 ± 0.09	7.37 ± 0.59	−4.5	*P* ≤ 0.05
PaO_2_	58.65 ± 4.87	79.29 ± 9.07	−20.0	*P* ≤ 0.05
PaCO_2_	50.35 ± 6.90	42.80 ± 5.35	15.8	*P* ≤ 0.05
Lac	3.34 ± 2.32	2.52 ± 1.77	7.1	*P* ≤ 0.05
EF value	47.53 ± 12.78	51.31 ± 10.45	−7.7	*P* ≤ 0.05
NT-proBNP	8074.15 ± 5464.43	6328.04 ± 4550.46	10.0	*P* ≤ 0.05

**Table 5:** The improvement of various indicators before and after treatment in the high-flow oxygen therapy group and the ordinary oxygen therapy group.

Project (difference before and after treatment)	High-flow oxygen therapy group	Normal oxygen therapy group	*t* value	*P* value
HR	15.5 ± 6.7	10.6 ± 4.3	46.9	*P* ≤ 0.05
RR	5.7 ± 2.4	3.3 ± 2.3	18.2	*P* ≤ 0.05
MAP	14.6 ± 9.9	10.7 ± 6.1	10.8	*P* ≤ 0.05
SaO_2_	9.9 ± 6.5	7 ± 3.4	13.1	*P* ≤ 0.05
pH value	0.071 ± 0.048	0.058 ± 0.038	25.4	*P* ≤ 0.05
PaO_2_	24.5 ± 11.3	20.6 ± 7.7	11.4	*P* ≤ 0.05
PaCO_2_	9.0 ± 7.7	7.6 ± 3.5	20	*P* ≤ 0.05
Lac	1.3 ± 1.2	0.8 ± 0.9	15.9	*P* ≤ 0.05
EF value	10.1 ± 6.2	3.8 ± 3.6	7.1	*P* ≤ 0.05
NT-proBNP	3920.1 ± 4566.1	1746.1 ± 1290.3	7.7	*P* ≤ 0.05

## Data Availability

The data used to support the findings of this study are available from the corresponding author upon request.
